# Efficacy and Safety of *Clinacanthus nutans* Lindau Cream vs. Podophyllin for the Treatment of Adults with Condyloma Acuminata

**DOI:** 10.1155/2022/1577716

**Published:** 2022-06-23

**Authors:** Sukhum Jiamton, Pattriya Chanyachailert, Yanisorn Nanchaipruek, Nuttagarn Jantanapornchai, Poramin Patthamalai, Pichaya Limphoka, Ya-Nin Nokdhes, Jiraporn Jantaravinid

**Affiliations:** ^1^Sexually Transmitted Disease and HIV Division, Department of Dermatology, Faculty of Medicine Siriraj Hospital, Mahidol University, Bangkok 10700, Thailand; ^2^Department of Biochemistry, Faculty of Medicine Siriraj Hospital, Mahidol University, Bangkok 10700, Thailand

## Abstract

Human papillomavirus (HPV) infection causes condyloma acuminata (CA). Podophyllin is the standard treatment. *Clinacanthus nutans Lindau* (*C. nutans*), a medicinal plant, has potent anti-inflammatory and antiviral effects. *C. nutans* cream is widely used in Thailand to treat the herpes simplex virus. We proposed that *C. nutans* might also induce CA clearance. There are no studies of *C. nutans* treatment of CA. This randomized controlled trial at Siriraj Hospital, Thailand, was conducted between January 2018 and December 2019. CA samples were obtained from 10 men with at least two CAs 1 centimeter apart. Each wart was randomized to a 4-week treatment with either *C. nutans* or podophyllin. The participants were 24 to 72 years old. Most HPV types were low-risk HPVs (HPV 11, HPV 6). Median CA clearance with podophyllin was a 97% CA clearance with podophyllin and 82% with *C. nutans*. *C. nutans* may be an alternative treatment for CA.

## 1. Introduction

Human papillomavirus (HPV) is the most common sexually transmitted infection worldwide [1]. More than 200 types of HPV have been identified [2]. They can be subdivided according to their oncogenic potential into high-risk (HR) or low-risk (LR) types. The immune system clears most HPV infections within 2 years of onset, and persistent HPV infection is essential for tumorigenesis, transformation, and progression [3]. HR types are strongly associated with malignant diseases such as cervical, anogenital, and oropharyngeal cancers [4], while LR types, such as HPV 6 and 11, are detected more frequently in condyloma acuminata (CA) [5]. HPV induces hyperplasia and hyperkeratosis, which are present clinically as warts [6].

CA has a significant impact on the quality of life [7]. Its treatment is usually lengthy and painful. Most current treatment options work by destroying affected tissues. The options consist of cytotoxic therapies (trichloroacetic acid, podophyllin, and 5-fluorouracil) or physically ablative therapies (cryotherapy, carbon dioxide laser, electrodesiccation, and surgical excision) [8, 9]. The location and number of lesions and the cost of treatment are considered when determining the extent of the therapy required for a patient.

Podophyllin is a plant-derived compound that causes tissue necrosis by arresting cell division and mitosis. Podophyllin may be applied directly to CA once a week, and it should be washed off 4 hours after treatment. The purified form is preferred as it has a good safety profile [10].

Clinacanthus nutans Lindau (*C. nutans*) is another herb belonging to the Acanthaceae family and is used as a well-known herbal medicine. In Malaysia, Indonesia, Thailand, and China, the plant is used as an alternative medicine for insect bites, skin rashes, herpes simplex virus (HSV) and varicella-zoster virus infection, diabetes, and gout [11, 12]. Because several experiments have reported antiviral activities, *C. nutans* is also recommended as an antiviral agent against HSV and VZV [13–15]. *C. nutans* has biological properties, such as antioxidant activity, antiviral activity, anti-inflammatory activity, and immunomodulatory effects [16]. *C. nutans* is safe as *in vivo* study on the toxicity of *C. nutans* did not show any toxicity [12].

In Thailand, *C. nutans* cream has been approved by the Thai Ministry of Public Health and is available in the market. To our knowledge, there is no study on the effectiveness of *C. nutans* cream for CA treatment. Our objective was to compare the efficacy of *C. nutans* and podophyllin for the treatment of HPV-infected CA by determining the CA size reduction in Thai males.

## 2. Materials and Methods

### 2.1. Study Population

This randomized controlled trial enrolled Thai men between January 2018 and December 2020. The inclusion criteria were as follows: (1) Thai men attending the Sexually Transmitted Disease Clinic at Siriraj Hospital; (2) 18 years or older; (3) willing to participate and give their written consent; (4) a diagnosis of anogenital warts by clinical manifestation; and (5) the presence of at least two CAs that were 1 centimeter apart. The exclusion criteria were as follows: patients (1) with HIV, (2) taking immunosuppressive drugs, or (3) with an autoimmune disease.

#### 2.1.1. Product

1. Podophyllin was produced by Vidhyasom Co Ltd, Bangkok, Thailand. The concentration was 25% podophyllin which constitutes of podophyllum resin 25 g in compound tincture of benzoin 100 ml.
2. *C.nutans* cream was produced by the Government Pharmaceutical Organization (GPO), Bangkok, Thailand, and the Thai Ministry of public health has approved *C. nutans* cream on the National list of essential medicine. The constitution was *C. nutans* extract powder 4.343 g in cream 100 g.

#### 2.1.2. Procedure

Before starting its trial, its protocol was approved by the Siriraj Institutional Review Board of the Faculty of Medicine Siriraj Hospital (approval number 550/2559 [ECI]). Written informed consent was taken from the eligible patients, and questions were asked and clinically evaluated. Their medical history was taken, and a physical examination was performed. The lesion sites were the shaft of the penis, glans of the penis, neck of the penis, and glans of the penis. The participants were randomly assigned by a block of four. Specimens swabbed from lesions in the genital area were collected and kept in cryopreserved tubes at −80°C. HPV genotyping was performed by the linear array HPV genotyping test (Roche Diagnostics, Switzerland), based on a reverse hybridization of amplicons to immobilize membrane-bound probe. HPV DNA in the swabbing sample was detected by multiplex PCR targeted to amplify the conserved L1 region of the viral genome. The system involves coamplification of the *β*-globin gene as an internal control. The PCR, performed in a 100 *μ*L reaction volume, was composed of a 50  *μ*L linear array master mix and a 50 *μ*L of DNA, as per standard protocol. After amplification, the biotinylated-PCR products were denatured immediately by adding 100 *μ*L NaOH to each PCR tube. Hybridization of the denatured amplicons and genotyping were performed on the GT-Blot 48, as per the manufacturer's instruction. Only samples that give a positive signal for *β*-globin were considered for analysis. Using the linear array HPV reference guide, the strips were manually interpreted using the linear array HPV reference guide, by reading the individual types down the length of the strip. The 37 HPV types that were analysed for comprised 13 HR-HPV types (16, 18, 31, 33, 35, 39, 45, 51, 52, 56, 58,59, and 66) and 24 LR HPV types (6, 11, 26, 40, 42, 53, 54, 55, 61, 62, 64, 67–73, 81–84, IS39, and CP6108). Genital wart samples in one patient were randomized in a block of four to separate genital warts as A and B. Each wart was randomized for treatment with either *C. nutans* or podophyllin. The participants received *C. nutans* as a home remedy and were instructed to apply the cream 4 times daily. Follow-up appointments were scheduled for each week for 4 weeks. Wart sizes were measured at each of the 4 follow-up sessions.

### 2.2. Statistical Analysis

Statistical analyses were carried out using PASW Statistics for Windows, version 18.0 (SPSS Inc., Chicago, IL, USA). The mean, standard deviation, mode, median, maximum, and minimum were analyzed and reported as percentages. Pretreatment and posttreatment values for podophyllin and *C. nutans* were compared using nonparametric Wilcoxon signed-rank tests and paired t-tests. Statistical significance was accepted for *P* values less than 0.05.

## 3. Results and Discussion

### 3.1. Results

The ages of the 10 male participants ranged from 24 to 72 years, with a mean (SD) of 38.7 (16.2) years.  Table 1 details the demographic data of the participants. Half were single, 40% were married, and 10% were divorced. Approximately 40% of the participants reported having a vocational education. Sixty percent of the participants were business owners. Only 20% of the participants had an underlying disease (allergic rhinitis in all cases). All participants had had multiple partners in their lifetime, had their last sex during the previous 6 months, and sometimes used condoms. Regarding sexual orientation, 90% reported being heterosexual, and 10% reported being bisexual. Twenty percent of the participants had a history of other sexually transmitted diseases.

All participants (100%) were HPV positive. There were both low- and high-risk HPV types. Mostly, the HPV types were HPV 11, followed by HPV 6. Approximately 50% of the patients were coinfected with multiple types of HPV, and 40% had multiple genital warts (Table 2).There was no specific clinical difference between the HR-HPV group and the LR-HPV group.

At the end of the treatment course, 9 patients showed more than a 75% reduction in CA lesion size, compared to baseline, with podophyllin treatment. Three out of 10 patients (ID 01, 05, and 10) achieved a 100% reduction with podophyllin treatment. Regarding *C.nutans* treatment, 6 of the 10 patients showed a more than 75% reduction, but only 1 patient completed the treatment with a 100% reduction (Table 3 and Figure 1).

The median total clearance for the podophyllin treatment was 97% CA reduction due to the CA clearance. However, the median total clearance for the *C. nutans* treatment was an 82.5% CA reduction (Table 3). There was a statistically significant difference for podophyllin treatment over *C. nutans* treatment (*P* < 0.001).

## 4. Discussion

CA is a benign disease caused by LR HPV. Our study showed that the most common types of HPV in CA were HPV 6 and 11. This result is consistent with the previous studies in Thailand, the United States, Brazil, Mexico, and China [17–20]. We also found that coinfections with multiple types of HPV were frequent, which is in agreement with prior studies [21].

To our knowledge, this was the first controlled clinical trial to compare the efficacy of podophyllin and *C. nutans* in clearing HPV-infected CA. We evaluated the efficacy of the 2 treatments using 10 patients.

Treatments for CA include topical therapies applied by the patient or the clinician and cytotoxic or physically ablative therapy approaches. Recurrence rates have been reported to range from 25% to 67% [22]. One-third of patients have been reported to clear spontaneously [23]. In Thailand, patient-applied treatment is imiquimod, and clinician-applied methods are podophyllin, trichloroacetic, cryotherapy, carbon dioxide laser, electrosurgery, and surgical excision. Currently, evidence for more effective alternative treatments is limited. Another consideration is that the costs of the various treatments available differ markedly. According to an evidence-based review, the first-line destructive treatment is cryotherapy, but the more expensive surgery and electrodesiccation options are more effective than cryotherapy. Similarly, first-line topical treatments are currently podophyllin and imiquimod [22]. However, since imiquimod is expensive in Thailand, we prefer to use podophyllin.

Podophyllin is derived from the roots of the mayapple plant (*Podophyllum peltatum*). Podophyllin is a cytotoxic agent that binds to the tubulin subunit of spindle microtubules and arrests mitosis in metaphase, eventually disrupting viral activity [24].The use of podophyllin is an effective, safe, and noninvasive method for CA treatment. In randomized controlled trials, podophyllin yielded moderate clearance rates of 41% to 77% and surprisingly high recurrence rates between 25% and 70% [25]. The side effects of podophyllin include local skin reactions and the potential for systemic absorption, including neurological toxicity, bone marrow suppression, teratogenicity, mutagenicity, and death [26]. Pregnancy is an absolute contraindication to treatment. Due to its adverse effect profiles, podophyllin should be treated with provider-administered treatment. However, podophyllin is still used for the treatment of CA due to its easy availability [27].

*nutans* is a medicinal plant known as “Praya-yo” in Thailand. It has been reported to have anti-inflammatory, antiviral, antimicrobial, and antivenom activities [28]. In Thailand, it is a well-known treatment for the herpes simplex virus, and the cost of treatment is reasonable. Limited evidence from a systematic review and meta-analysis of randomized clinical trials showed some beneficial effects of *C. nutans* preparations for treating herpes genitalis [29]. In Thailand, the GPO of the Ministry of Public Health produces 4% *C. nutans* cream for patient-applied treatment. The medication is applied 4 times daily.

This study evaluated the effects of treating HPV-infected CA with podophyllin (the gold standard; applied weekly by doctors) and 4% *C. nutans* cream (applied 4 times daily by patients). The clearance rate of the podophyllin treatment was noticeably higher than that reported by an earlier study [30]. As to the *C. nutans* treatment group, the clearance rate was lower than that of the podophyllin group for all patients.

However, the efficacy of the *C. nutans* treatment was lower than that of the podophyllin treatment. We suggest combining both to treat CA, for example, having patients apply *C. nutans* cream at home every day and visit their doctor weekly for podophyllin treatment.

Some limitations were in our study. First, as there was a small sample size, a larger cohort is needed to validate the optimal dosage of *C. nutans* for the treatment of CA. Furthermore, the recommended application of *C. nutans* cream 4 times a day for an HPV infection may not be convenient or practical for some patients.

## 5. Conclusions

Our study found that *C. nutans* may be beneficial for the treatment of CA. *C. nutans* may be used as an adjuvant treatment for CA.

## Figures and Tables

**Figure 1:** Condyloma acuminata on corona of the glans penis (ID 02) was treated with podophyllin and *C. nutans* for 4 weeks, with a resulting condyloma acuminata reduction. (a) Prepodophyllin treatment. (b) Postpodophyllin treatment. (c) Pre-*C. nutans* treatment.(d) Post-*C. nutans* treatment.

**Table 1:** Demographic data of participants.

	*N* = 10
Mean (±SD), range (years)	38.7 (16.19), 24–72
Marital status	
Single	5
Married	4
Divorced	1
Education	
Primary	1
Secondary	2
High school	2
Vocational	4
Bachelor's	1
Occupation	
Government officer	2
Business owner	6
Business officer	2
Having multiple partners	10
Sexual orientation	
Heterosexual	9
Bisexual	1
Contact with sex workers in last 5 years	2
Having tattoo	3
Smoking	2
Alcohol drinking	7
Having sex within last 6 months	10
Intravenous drug use	
Used in the past	1
Current use	0
Condom use	
Always	0
Sometimes	10
Never	0
History of STI	
Yes (gonococcal infection)	2
No	8

STI, sexually transmitted infection.

**Table 2:** Details of genital warts and HPV^Ɨ^ genotyping of each participant.

Patient (no.)	Age (years)	Lesion sites	HPV genotyping		Number of lesions
			Low-risk	High-risk	
01	25	Shaft of penis	6	—	Single
02	58	Corona of glans penis	11, 40	—	Multiple
03	44	Shaft, neck, and glans of penis	11, 81	45, 58	Multiple
04	24	Shaft of penis	6	—	Single
05	45	Shaft of penis	6	—	Single
06	28	Glans of penis	11	—	Single
07	32	Corona of glans penis	84, CP6018	16	Single
08	72	Shaft of penis	11, 51	54	Single
09	33	Corona of glans penis	6, 62, C6108	51, 58, 59	Multiple
10	26	Glans of penis	11	—	Multiple

^Ɨ^HPV, human papillomavirus.

**Table 3:** Comparison of CA^Ɨ^ dimensions and percentage reductions for podophyllin and *C. nutans*^ǂ^ treatments.

Case no.	CA dimension in millimeters					
	Podophyllin treatment			*C. nutans* treatment		
	Pretreatment	Posttreatment	(%) reduction in size of CA	Pretreatment	Posttreatment	(%) reduction in size of CA
01	20 × 5 × 3	No lesion	100	10 × 5 × 3	No lesion	100
02	10 × 10 × 3	3 × 3 × 1	97	20 × 5 × 5	5 × 3 × 3	91
03	30 × 20 × 10^a^	20 × 16 × 8^b^	70	30 × 20 × 10^c^	25 × 20 × 10^d^	50
04	3 × 3 × 2	1 × 1 × 0.5	97	3 × 5 × 3	2 × 4 × 1	87
05	2 × 3 × 2	No lesion	100	2 × 3 × 2	1.5 × 1 × 1	82
06	2 × 2 × 2	1 × 1 × 1	87	3 × 5 × 3	2 × 3 × 2	73
07	5 × 5 × 5	2 × 2 × 1	97	5 × 5 × 2	2 × 2 × 1	92
08	5 × 15 × 5	2 × 2 × 1	99	10 × 10 × 2	8 × 8 × 1	68
09	2 × 2 × 2^e^	2 × 2 × 2^f^	96	2 × 2 × 1	2 × 0.5 × 1	75
10	1 × 2 × 2	No lesion	100	2 × 2 × 3	1 × 1 × 2	83
	Median (min-max)		97 (70–100)	Median (min-max)		82.5 (50–100)
	Mean ± SD		94.3 ± 9.36	Mean ± SD		80.1 ± 14.32

^a^, 14 lesions;^b^, 10 lesions;^c^, 15 lesions;^d^, 9 lesions;^e^, 5 lesions;^f^, 4 lesions; ^†^CA, condyloma acuminata; ^ǂ^*C. nutans*, *Clinacanthus nutans* Lindau.

## Data Availability

The data used to support the findings of this study are available from the corresponding author upon request.
